# Using Blockchain Technology and Sharing Culture to Promote Sustainable Forest Management in Tribal Communities

**DOI:** 10.1155/2022/1529407

**Published:** 2022-06-30

**Authors:** Yixiao Peng, Wenyi Huang

**Affiliations:** ^1^School of Economics, Zhejiang University of Technology, Hangzhou, China; ^2^Postgraduate Programs in Management, I-Shou University, Kaohsiung, Taiwan

## Abstract

Forest protection is crucial to ensuring the balance between human beings and ecology. This study explores the key role played by communities that originally lived in forest-protected areas in implementing the traditional management of forests. The unified management mode previously used by the state power can no longer meet the demands of modern times; hence, multiple types of management systems should be implemented to enable adaption to the original ecology of forest areas. A multimodal management mode should be adopted to restore the original ecology of forest areas. The adoption of this management system can restore a forest to its original state (i.e., the state that existed prior to the entry of state power). The forest has been in a state of ecological balance involving numerous species since ancient times. However, in the modern field of science, the passive restoration of a community's self-governance ability could be unsustainable and unstable. To improve this situation, blockchain technology can first be used to improve the community management of a forest, such that the capabilities of the original local community can be improved; second, tourism promotion benefits both the community and the forest. When a community in a forest develops the tourism industry with the support of blockchain technology, the information and resources of all parties can be widely connected with the larger world, and this considerably increases success rates; finally, the traditional spiritual culture of a community, such as the culture of sharing, should be promoted. In addition to the skillful utilization of technology, culture can improve the traditional forest management ability of tribal communities who live in native forest areas in terms of their personality traits. Overall, we conclude that: against the evolution history of the over one hundred years, the adoption of new technology for forest management is inherently a creative innovation for the tribal community's entrepreneurial development.

## 1. Introduction

Tribal communities living in the forest have maintained a state of balance with the ecology of the forest since ancient times, just like the other species that live in the forest. This balance was not broken until the interference of an external force, namely the power of the state. The main purpose of state interference is to obtain forest resources. Hence, many management models for obtaining resources have been developed. The acquisition of forest resources started with visible trees, minerals, and medicinal plants, which was followed by the introduction of land loss protection, air environment protection, and climate change stability policies; these are all direct or indirect means of acquiring forest resources.

Among the forest management strategies that were adopted by various countries for tribe communities located in forests, the first was the strategy of providing regional protection to an entire forest. When a management implements this decision, they adopt expulsion-oriented methods to forcibly move tribe communities out of protected areas. The second type of management strategy involves the adoption of a cooperative model in which the tribe community in a protected area is a participant, especially a tribe community that is based in the land around a forest or buffer zone. People who adopt the third type of management strategy believe that having the status of a protected area does not, by itself, ensure the effectiveness of conservation policies. Instead, they assert that people should gradually adopt multiple forest management strategies, including the integration of people in a community area as management participants [1].

The intrusion of state power in the development of forest resource management strategies and planning has resulted in poor execution results in numerous forest reserves, forcing policymakers and scholars to reconsider the utility of communities in resource utilization and conservation [2]. The main reason for incorporating community participation into strategic forest management is that traditional knowledge is acquired by local people through the accumulation of experience and informal experimentation and the development of a deep understanding of the environment in a specific cultural context. Traditional knowledge can become social knowledge, facilitate communication and decision-making, and serve as a management basis for local institutions [3].

First, although community participation is gradually being incorporated into forest management, comprehensive policy-related assistance has not yet been provided. Consequently, communities often cannot fully restore their long-standing management habits in relation to forests [4]. Second, communities living in forests do not consider the improvements to their quality of life. Hence, they move out of the forest areas that they grew up in because of distress and do not consider the long-term development of their tribal community in the forest [5]. Third, no study has thoroughly discussed the influence of a traditional community culture on forest management [6]. Fourth, modern science and technology have not been applied to study the original forest management abilities of original forest-dwelling communities and assist tribe communities in identifying appropriate and innovative modern technological methods during the process of social transformation, such that the traditional forest management abilities of tribal communities can be effectively preserved [7].

Through the present study, the researchers aim to: (1) discuss the feasibility of a new partnership between the Paiwan tribe community and national policies, (2) utilize blockchain technology to support the re-development of the traditional management ability of the community, and (3) leverage the local culture of sharing such that management rules can be internalized in the personality traits of community residents and concrete suggestions relating to community forest management can be proposed.

## 2. Literature Review of Forest Protection History

### 2.1. Evolution of Forestry Management in the Paiwan Tribe Community

After it lost the Sino-Japanese War in 1895, the Qing Dynasty was forced to sign the Treaty of Shimonoseki to confirm its cession of Taiwan and Penghu to Japan. The regimes of the various islands of Taiwan gradually started to enter a state of comprehensive management at the national level. Previously, power at the national level did not have an effective presence in various areas in the islands of Taiwan. Therefore, the indigenous Paiwan tribal community adopted the forest management mode that was handed down to them from ancient times through living culture. Most indigenous people live in high mountains, and their traditional living areas are divided into forest hunting, farming, and community residential areas. The utilization of forest areas usually involves entering a forest to gather fruits and plants or to hunt in accordance with seasonal or ritual practices; it also involves entering a forest area to obtain the wood materials required for the construction of community houses. These activities, which involve visiting forests, are temporal, regional, and purposeful, and the tribe residents will not dwell or gather resources in a mountain forest for a prolonged period without a specific purpose. The members of the tribal community are warned against straying into certain areas, or they will be punished by divine powers. Therefore, some forests are regarded sacred forests, and the amount of edible fruits that can be picked from these forests is limited. For some areas, specific groups are assigned to manage them and ensure that the tribe community does not lack rain and water sources. The groups with this responsibility protect forest resources and are similar to law enforcement officers [8, 9].

The entrance of Japan into Taiwan marked the intrusion of state power into the Paiwan tribe community. State power forcefully dominated the rules of life and cultures of all tribal communities, and all of the forests in traditional regions were nationalized. The hunting quotas and seasons were stipulated by the Japanese police, the method of farming changed from burning and rotational cultivation to fixed farming, and the ownership of the land by a tribal community was redistributed from the chieftain level to individuals under a private property system. A clear distinction is made between agricultural farming land and forest land. Consequently, the area of farming land was considerably reduced, and hence existing farming lands were used more frequently. The state power then did not regard the crisis of environmental ecological imbalance as a focus of their governance. Instead, they focused on suppressing the rise of rebellions in tribal communities. The Paiwan tribe underwent a community reconfiguration at that time; a relatively flat area with a small slope was selected to forcibly combine all the surrounding small tribal communities into a large community with approximately 300 households to facilitate the management and implementation of life culture education. Orally transmitted knowledge is generally local, collective, experiential, and holistic. Therefore, memory is the key intellectual resource in tribal community culture [10].

After losing the link with land management and the free environment of transmission, the tribal community's ability to manage forests was almost completely removed at that time. The original autonomous structure of the tribal community could no longer function, and the original ecology balance mechanism that was based on forests and tribal communities ceased to exist. Fortunately, the Paiwan tribal community is located in Taiwan, which has a tropical monsoon climate; most of the forests that were located close to the community had no precious trees, and only a few of them were stout camphor forests. The impression of the local people was that the Japanese government did not conduct large-scale forest resource exploitation that affected the Paiwan tribe.

In 1945, the Empire of Japan withdrew from Taiwan entirely. With regard to the management of the indigenous people in Pingtung County, the succeeding government continued the model used by the Japanese government to calm rebellions. For tribal community management, the principle of centralized management was adopted. Furthermore, the collective migration of the tribal community to the hilly forest zone near the plain area, which was originally planned by the Japanese government (1), was carried out by the succeeding government. The justifications for this migration included the dangerous terrain and barren soil conditions in the mountainous area that the community lived in and the difficulties in improving agricultural management, transportation, and living facilities. In summary, the government exercised its power to move indigenous communities out of the alpine forest areas that they had been living in for a long time. Through various means such as semi-oppression, subsidies, and incentives, numerous indigenous tribe communities were persuaded to move out of their original living areas, which they had lived in for hundreds of years or even longer. Under these circumstances, the Paiwan tribe community gradually moved to a hilly woodland that was located near a plain in 1976.

However, because the new area did not contain public arable land, such that the ownership of arable land in the traditional regions could not be proportionally converted (in terms of land area) into ownership of arable land in the new area, the strategy adopted by the government was to relocate the residential area of the tribal community while retaining and reserving the arable area in the original living area for the tribal community. At that time, the forest area where the community was located was completely owned by the state and subjected to an expansion. During the process of land privatization, the area owned by individuals was limited.

### 2.2. Relationship between Land Management and Forest in the Paiwan Tribal Community

If the forest is located within the traditional territory of a tribal community, community members can use forest products in accordance with their traditional customs. However, after a tribal community is separated from its land, their access to the forest is greatly reduced [11]. Additionally, a few residents still lived self-sufficient lives in the traditional regions of the tribe by engaging in traditional crop farming, hunting, and medicinal plant gathering. With a sparse population, the area of cultivated land decreased. Given that large areas of land had been abandoned for a long time, the forest area naturally expanded, and the cultivated area was gradually taken over by forest trees. After approximately 20 years of recuperation, the trees in the forest have grown into towering trees. In this environment, where people, animals, and plants have lived together for thousands of years, the roles played by tribe community residents in ecological balance have gradually disappeared following the implementation of the national relocation policy. The culture produced through the interactions between the tribe community and the environment has also diminished accordingly.

After 1990, businessmen in the wood industry identified a business opportunity involving the deforestation of private land and negotiated with private landlords to purchase trees from such lands for farming and animal husbandry. For a period of time, numerous deforestation projects were conducted in the traditional regions of the tribal community, and the government also granted approval for deforestation on the basis of loose guidelines.

During the decades of deforestation, no one in the tribal community cared about how their land could be utilized after deforestation because of the economic benefits that they gained from deforestation, even though these benefits were limited. With this highly passive attitude, the tribal community residents were expecting weeds and pioneer tree species to grow naturally. They were apathetic about the loss of land due to heavy rain. Instead, they were happy with the limited income that they received. Because most tribal community residents have moved to cities and towns to work as low-level laborers, interactions between the community and their land were limited. Furthermore, the residents had no economic incentive to utilize their land. This situation continued until the forests were fully deforested. The government was also alarmed by the severity of the deforestation problem after they found out that the land in the traditional regions of the tribal community was full of excavated and cleared surfaces. Hence, they began to strictly restrict the deforestation of private land [12].

Similar to how other resources with direct value for humans are protected, the conservation of forest resources involves a complex socio-ecological system; therefore, prudent decision-making is required [8]. Initially, tribal community residents did not understand why the government introduced the private land logging prohibition policy. Moreover, when the tribal community moved to the woodlands on the hills, there were no or only a few trees on the agricultural lands in the mountains where they used to live in; following the subsequent cessation of farming, trees grew naturally on these lands, and these trees attracted timber merchants to purchase them and acquire economic benefits, which was a positive development for the landlords.

However, the tribal community residents' unfamiliarity with the land that they moved to prevented them from understanding the various land protection measures that their tribespeople previously implemented in their traditional territory. These measures included the tribal community's rigorous flood control facilities for land management that were built when they were farming in traditional territory, i.e., the construction of each slope involved layers of terraced rocks that were placed to block heavy rain and floods, such that direct and strong scouring to the topsoil can be prevented. Recent scientific research has revealed that terraces not only stop water flow but also prevent soil erosion [13]. Therefore, in terms of overall landform, their cultivation over the past hundred years has not caused large-scale rain erosion leading to land loss. Arguably, the tribal community's land management was integrated into the ecology as a whole and played a role in balancing it; human habitation did not alter the land strata or disrupt the balance of existence of surrounding species.

Lawler stated that the government's willingness to help enables the sustainable development of tribal community forestry; the second factor for such development is meaningful timing, adequate deadlines, environmental safety, and most crucially, the decentralization of governance responsibilities [14]. Therefore, if the government had interacted with the community while taking into account the aforementioned factors, it probably could have increased the community's willingness to cooperate with respect to the relevant policy amendments and learn more about the traditional knowledge for maintaining a balanced relationship between the local community and the trees; consequently, the poor communication with the tribal community during the government's implementation of policy changes (i.e., shift from the authorization of deforestation by timber merchants to the complete ban on deforestation) could have been avoided. Furthermore, the tribal community would not have been displaced from their traditional territory because of the government's persistent implementation of village relocation in the early years, which gradually reduced the tribal community's ability to undertake independent forest management and exposed them to unpredictable external impacts, allowing timber merchants to completely deforest the traditional territory where the community had lived in for an extremely small profit. Because of the government's failure to adequately consider the community's rights and interests, negligence in developing its ability to restore traditional self-management, and disregard for other methods involving multiple-use forest management, the damage to the trees and lands of the community persisted, leading to the unfortunate failure of the tribal community, which had resided there for thousands of years, to maintain local sustainable development.

### 2.3. Effect of Government Forest Management on Tribal Community Management

Direct payments for ecosystem protection are increased in popularity because of their high effectiveness; specifically, it is more targeted and conditional, especially for governments that lack effective command and control measures [5]. Therefore, the government proposed a two-stage forest protection policy after recognizing the crisis pertaining to the country's overall territorial security, which was associated with its arbitrary approval of deforestation proposals and the large-scale deforestation of private forest lands.

The first-stage forest protection policy stipulates a ban on deforestation in catchment areas and the granting of subsidies through an afforestation subsidy policy.

The second-stage forest protection policy subsidizes the complete ban of deforestation on private lands.

The two stages of the aforementioned subsidization policy attained and even exceeded the subsidization goal set by the government. Specifically, the second stage was more popular than the first. Applications were made for almost all the land categories pertaining to forest land. Moreover, some landowners attempted to obtain more subsidies and applied for land use change, which converts the status of agricultural and pasture land with trees into that of forest land, to facilitate their subsidy applications. Under the current laws and regulations, such changes are considerably difficult to reverse once they are made. Consequently, the conversion of large plots of agricultural and pasture lands into forest lands restricted the legitimization of farm land, which increased the alienation of the tribal community residents from their lands, especially for the next generation of landowners whose lives were primarily based in towns. These residents were only concerned about the subsidies for afforestation and the ban on deforestation, and they lacked a clear understanding of the location or current forest growth of their lands. At that point, the government had attained its goal of afforestation, but the initial tribal community residents were distanced from their lands, leading to their negligence of land management, which caused unforested agricultural and pasture lands to fall into disuse. No remedies or improvements were proposed to address this problem. Meanwhile, the culture, living habits, and oral history of the indigenous community residents in relation to their lands were disappearing rapidly. The distancing is such that they held feelings only for the original relocated sites and only regarded the surrounding private forest lands and agricultural and pasture lands as sources of subsidies for afforestation and the ban on deforestation. If this situation persists, the original tribal community residents will inevitably disappear from their traditional territories [15]. Forests are home to most of the tribal communities and minorities worldwide. In fact, forests are crucial for tribal communities because the forests that they inhabit provide them with the necessities of life (e.g., food and water) and enable them to form cultures, engage in recreational activities, and build their histories. Through their extensive experience with respect to forest life, tribal communities have developed an impressive foundation of practical knowledge regarding their environment. When it is managed properly, this knowledge can be employed in forest policy formulation, conflict resolution, sustainable natural resource management, and the development of novel technologies to achieve enhanced results [16–18].

### 2.4. Effect of Opening Up to Tourism on Communities' Forest Management

The actual relations between tribal communities and the natural environment are highly diverse; such relations vary in terms of social and customary aspects and among locations. With a social hierarchy that is diversified and provides a sense of belonging, indigenous tribal peoples may hold greater respect toward their local environment than most societies because of their close bonds to their ancestral lands, their common system of property management, and their awareness of land trusteeship for future generations [19]. Therefore, the sustainable development of tribal communities is a challenge that requires an immediate solution.

Over time, the government of Taiwan lifted entry restrictions to mountainous areas and loosened approval requirements for entry into most mountainous areas. Moreover, the service industry formed a general trend among Taiwan's industries, and the number of leisure activities held in mountain forests gradually increased, particularly after the 2-day weekend was fully implemented in Taiwan on January 1, 2001. Therefore, in line with the public's expectations, the government began to invest resources into developing mountainous areas.

To support the start-up tourism industry, the Paiwan Tribal Community Development Association acted as the leading organization. A working group was formed under the guidance of the chairperson of the association. Comprehensive assistance was provided by the township office and county government with respect to staff training, the restoration of on-site slate houses, and the construction of public facilities. Moreover, the Maolin National Scenic Area Administration (MNSAA) later designated the area as a site that would receive prioritized tourism promotion guidance. Negative effects also emerged with the increase in tourist numbers; they included concerns about safety and hygiene in the context of the incomplete infrastructure of the tribal community. Additionally, with easy access to the site and the surrounding mountains and forests, some tourists began to perform illegal acts such as randomly collecting precious forest trees, plants, and minerals on the mountains; hunting animals and centipedes; and even arbitrarily occupying public and private land to facilitate frequent visits to leisure areas.

Some travelers relied on their extensive legal knowledge and favorable media relations to assert that transportation facilities, mountains, and water are all public goods that should be shared by all citizens, i.e., no one should be prohibited from accessing these areas. When the tribal community did not comply with the demands of these travelers, these travelers called in the media to cover this news. The descriptions and texts accompanying the broadcasted images were highly offensive, with statements such as “What era are we living in? Why are there people who act like kings of their mountain fortresses in Taiwan? They forcibly occupy and claim forest resources.”

Given the key role of tribal communities in the conservation of biodiversity, local community empowerment must be recognized. This is an opportunity for the tribe to steadily enhance their territory and natural resource control and obtain full access to relevant information and technology. Notably, legal and enforceable rights related to land and water provide communities with economic incentives and a legal basis for governance [10]. Therefore, the Majia Township Office recently implemented the demarcation of natural and cultural scenic areas, and applied to the Pingtung County Government for approval to designate the road leading to the Paiwan and Makazayazaya tribal communities as a township-level fifth special road Sisaumaqa Djalan with regulated access in accordance with local self-governing provisions. However, at the time of writing, the related enforcement methods are still undergoing modifications.

Meanwhile, the forestry-related government agencies were ineffective in controlling access to mountainous areas because numerous visitors entered them via the open entrance of state-owned mountainous areas, and the insufficient number of patrolmen has prevented the enforcement of mountainous area access control regulations relating to entry permit requirements.

Tribal communities face explicit and implicit oppression with respect to their traditional territories [20], and they generally fail to implement successful ecotourism projects because of many factors, including isolation as well as the lack of financial resources, management skills, and infrastructure. The use of complementary economic instruments and promotion of the so-called charismatic endemic species may be key factors for maximizing revenue from ecotourism activities [4]. Therefore, challenges related to tribal tourism promotion must be overcome. In the past, the traditional territories of tribal communities were only used for self-sufficient agriculture, hunting, and food gathering. By contrast, tourism promotion provides tribal communities with a brand-new domain for survival and development, which induces interactions between traditional territories and the outside world. To generate economic benefits, the utilization of resources in the traditional territories by tribal communities is considered, allowing them to return to and live in these territories and to extend their feelings and cultures in relation to their lands.

## 3. Methodology and Sample

In the present study, a qualitative research design was adopted. The methodological foundation was from the intersection of Sociology and Politics and Anthropology. Since the issue we explored is a societal wide and complex issue for environmental protection (which is largely related to the special issue), and at the intersection of ethnic and governmental and technological imperatives, it is important to adopt a whole-oriented approach to cover as much concerns as possible. In the present study, the studied community's application of blockchain technology in forest management and tourism promotion was examined. The researchers attended the ministerial conferences, sacrificial ceremonies, and Church events held by the studied community and conducted in-depth interviews with community residents. These methods were adopted to understand the traditional forest management knowledge that the tribe had accumulated and the state of their blockchain information platform usage; they were also used to analyze the sustainable forest management practices of the studied tribal community.

The sample, Paiwan tribe community (the Paiwan ethnic group is an indigenous ethnic group in Taiwan, and the Paiwan tribe community has the same name as the Paiwan ethnic group), belongs to Taiwan's indigenous Paiwan ethnic group and serves as the subject of the present study. This community was selected mainly because its living area had changed tremendously during the process of modernization. The community was separated from the mountain forest that they live in by forceful eviction, and its tribal residents have been moving to cities and towns to make a living for decades because of social changes. These residents undertook basic labor work in cities and towns. Thus, the original mountain living habits and cultural traditions of these people have almost been fully forgotten. Because of Taiwan's economic growth in the past decade, the transportation and environmental infrastructures in traditional living areas (i.e., those that the aforementioned residents originally moved out of) have improved. This development has enabled community residents to live their lives between their traditional communities and current places of residence. Furthermore, modern technological developments such as blockchain technology can enhance a community's traditional community-building abilities. Blockchain technology can be used to integrate the surrounding resources of a community and create a common platform for demand and supply.

## 4. The Narrative Results and Analysis of Adopting Blockchain Technology

The forest is an area of high engagement with numerous stakeholders. They also contribute substantially to the climate and are crucial for sustainable development in terms of resources, biodiversity, and other factors. By contrast, for the forests of today, managerial decision-making is generally guided by top-down organizational processes in which only some stakeholders are involved; however, the stakeholders who are seldom or not involved in decision-making are still affected by the decisions that are made. At the same time, the process of digital transformations takes place in almost all domains; it provides new methods of engagement and demonstrates how people can secure their interests. In this context, blockchain technology must be introduced and promoted [21].

Blockchain technology provides value by sharing the transactions recorded in a ledger and providing secure and auditable information through the issuance of a verifiable and time-stamped record of transactions [22]. These transactions are verified through a process that is consistent with the consensus rules of a network. After a new record is verified and incorporated to a blockchain, multiple copies are established in a decentralized manner, thus creating a chain of trust [23].

Tribal community residents position themselves as the guardians or protectors of the environment, and they have undertaken activities aimed at restoring degraded ecosystems and preventing further ecological damage [20]. Tribal communities generally have an extensive knowledge and understanding of local flora, fauna, and ecological processes, which were accumulated through observation, practice, and cultural transmission across generations [18, 24]. For the conservation and sustainable management of ecosystems and species, community-based conservation is increasingly being recognized as a key global force [25]. Tribal community involvement in forest development and protection is now a core component of global sustainable development efforts. Indigenous communities are culturally and spiritually connected to the forests in which they reside, and traditional land rights and community participation in forest management form the foundation for their values and lifestyles [14].

Since the 1990s, numerous people-centered protection strategies have emerged under the influence of trends relating to democracy and human rights. They emphasize the role of local people as stakeholders in resource management (e.g., bottom-up approach and public engagement). The rationale for engagement is that local people not only benefit from participatory resource management but also contribute to sustainable natural resource governance. Among the discussed concepts, community-based natural resource management accentuates the key role of local participation in natural resource management, which has become the primary concept [26].

The long-term effects of the government's afforestation policy and village relocation programs have separated tribal communities from their original traditional territories and altered their lifestyles. These effects have considerably changed the land management model of tribal communities. Given the diversity of modern career options, traditional agriculture is no longer a practical means of earning money. In this situation, the tribal community residents appear to be gradually losing their original living skills and habits that enable them to coexist in harmony with the forest. Accordingly, the development of tourism provides an opportunity for the status quo to be changed. Therefore, in community forest management and the application of blockchain platforms, tourism development is held as a goal of sustainable development.

The MNSAA is a national-level agency that specializes in assisting local communities with tourism development. It is involved in infrastructure construction and provides guidance relating to tourism operations. For tourism promotion, in addition to infrastructure construction, tourism product marketing is a key focus of the MNSAA, which promotes beautiful local mountains, waters, and sceneries, thereby attracting people to visit the Paiwan tribal community's traditional territories for leisure activities. To enable people to quickly access tourism-related information on the MNSAA website, a blockchain platform was used to establish a connection with the tribal community, and this platform was combined with other networks and digital media.

In addition to national-level agencies, local governments have also demonstrated their commitment to tourism promotion. For example, Majia Township Office, a local government office, has promoted the implementation of policies regarding establishing special roads for tourism purposes combined with the centralized management of travelers. Specifically, all people traveling into the mountain must take a shuttle at the shuttle stops set up by the Office. The number of travelers allowed to visit the mountain is subjected to a quota, and the routes of travel are controlled to ensure that the quality of tourism activities is not compromised by overcrowding in the mountain, and that these activities can be restricted to specific sites. Accordingly, a blockchain platform may be established for shuttle schedules and visitor quotas to enable community members to provide tourism services and allocate administrative resources in an appropriate manner at an early stage, thereby preventing the waste of resources, improving waste management, and enhancing environmental protection.

With the assistance of the central and local governments, the Paiwan community applied a blockchain platform to fulfil the following aspects of management.

1. Informatization of stories about the forests and land: The first step of informatization is to compile and informatize all historical events and ancient myths in the realm of tradition, such that guides can quickly familiarize themselves with these stories. These stories are further categorized to facilitate the appropriate assignment of stories to guides on the basis of their expertise. These stories reveal the bonding between people and the land over the last hundreds and even thousands of years, and travelers may choose their guides and itineraries through a blockchain platform. Story compilation enables travelers to learn about the beautiful stories of the mountain and the traditions of the local community, and it also enhances the cultural identity and confidence of community residents.
2. Centralized management and informatization of private forests: The management of private forests has shifted from a laissez-faire model to the effective use of forests resources. Forests with sightseeing value are incorporated into travel routes, and information about these forests is uploaded to the blockchain platform. This allows travelers to learn about the features and the difficulty level of each hiking trail in the forests online and select a trail in advance on the basis of their physical conditions, which greatly improves their experiences in the forests.
3. Informatization of unique service items: Travelers who wish to experience deep travel and stay for a few days in the community can make arrangements to stay in local traditional stone slab houses that are more than 100 years old rather than in tourist accommodations in scenic areas (e.g., beautifully constructed chalets or high-end, exquisite concrete-based buildings). This arrangement allows travelers to experience how the community has integrated itself into the local ecosystem and made effective use of local resources while maintaining a respectful relationship with the environment in terms of their housing. The accommodation options are informatized and categorized at several levels; their capacity is defined; and their features are incorporated into the blockchain platform to provide a diverse selection of accommodation options.
4. Supply chain integration for food ingredients and catering services: Local food ingredients are used in the dishes prepared for travelers. This promotes the traditional cooking techniques of the Paiwan community and provides incentives for the community to use lands that are designated for farming and grazing purposes, which help to balance plant ecology and recreate the bond between the community members and their land [27]. Cioca et al. [27] argued that customers do not pay more or sacrifice quality, convenience, or their brand preferences for social enterprise products, indicating that they do not focus on social enterprises when making purchases and are instead more concerned with the product and its brand, comfort, and price. Accordingly, the intention of customers to purchase must be emphasized in the development of products of public interest. The Paiwan community has created a blockchain for food ingredients that includes the cultivation and harvesting of ingredients, the demonstration of suitable cooking techniques, and ingredients that go well together. The blockchain increases the transparency of the food products and allows travelers to decide on the combination of food ingredients that they wish to sample before making purchases in the community.

Hipwell suggested that the following six tasks must be completed to achieve sustainable development. (1) The scale of a development activity must be small enough such that the local community can manage it without external assistance. (2) Such an activity requires active participation by general and representative members of the community. (3) The activity must generate actual benefits for the overall participants. (4) The activity must lead to a fair and general (optimal) improvement in the quality of life of community members. (5) The results of the activity must contribute to environmental protection and preservation. (6) The activity must enhance the maintenance or improvement of the cultural environment of the community [20]. Sustainable development emphasizes environmental protection, and it helps to alleviate the worsening state of global warming and climate change [28]. Numerous communities hope to manage their forest resources in a more general manner and shift their focus away from wood materials [29].

The Paiwan community has long lacked the technical capacity and experience to market its products. For example, community members value the culture of sharing; they farm mainly to maintain self-sufficiency and to share resources with their friends and family, and they lack practical experience in a production model that aims to achieve economically feasible yields and supply for the market. Therefore, income from farming is generally low for community members, which naturally leads to a lack of experience in crop marketing. Furthermore, they are hesitant about complementing their own crops and handcrafts. For example, they are unlikely to say that they grow the best, most delicious, or freshest vegetables or fruits in their area; proactively market their products at the market or to vendors; or organize food sampling events for their crops. To address the community's disadvantage in marketing, a community network-based blockchain platform was established and connected with a governmental marketing aid to provide preorder services and facilitate horizontal and vertical marketing. The blockchain platform greatly benefits the community in terms of redeveloping agriculture in the traditional region and restoring their biodiverse forest environment.

## 5. Long-Term Effects of a Sharing Culture on the Community's Sustainable Development

Becker maintained that indigenous communities typically make common property decisions that balance individual and community benefits [3]. Three types of incentives motivate people to participate in voluntary organizations, namely material, solidary, and purposive incentives [30]. The Paiwan community has long valued the culture of sharing, which has helped the community to sustain and continue their bloodline in difficult and barren environments. In a self-sufficient scenario where no external resource is available, sharing is the best means to provide for the community because it facilitates adequate exchange and utilization of resources. For example, *mazazeliuliulj* (a traditional task assignment system that involves arranging the order of tasks according to their urgency, with community members taking turns to work on the most urgent task until it is finished before moving to the next task) is a common practice in the community that utilizes labor sharing to provide collective support to families who have the most urgent tasks to complete. *Mazazeliuliulj* enables labor-intensive work (e.g., harvesting and the building of stone slab houses) to be completed in an effective manner. In the traditional hunting culture of the Paiwan community, the hunters move in groups, and a successfully hunted animal is cut into multiple pieces and shared with specific community members such that the old, disadvantaged, women, children, and families who have endured tragic events can all enjoy fresh meat. Collective restraints are also realized through the sharing of control over specific resources, which allows all community members to issue warnings and report on violations of rules concerning controlled resources in any area of the community, thereby effectively preventing unauthorized entry into the forests during nonhunting seasons or nonritual periods. This practice provides the local flora and fauna with adequate time to grow and reproduce and thus prevents the deterioration or loss of forest resources.

With the culture of the community serving as a foundation, sustainable development education can be implemented to encourage community members to respect lives, care for the Earth, and care for the Earth's community of life. These concepts are closely associated with the fundamental value of sharing, the principles of bioethics, and the knowledge of sustainable development [31].

A sharing culture should be promoted in everyday life and education to facilitate the centralized management of all travel routes in the promotion of the use of forest resources for tourism. Specifically, the potential effect of tourism on the mountain environment can be effectively controlled to allow for the sharing of sightseeing resources among all community members and prevent free competition among individuals [32]. Such free competition may encourage everyone to develop their own secret forest trails in an unrestrained manner; the use of such trails generates man-made waste that would be disorderly scattered across the forests and thus affect the environment and the growth of organisms.

## 6. Using Contemporary Scientific Methods and Equipment to Enhance the Community's Ability to Manage Forests

Community members have achieved a balance between their lives and the surrounding forest environment through their long-term interaction with it, and thus they have their own practices and experience with respect to sustainable forest management and development. However, this experience is challenging to apply or passed on. Accordingly, contemporary management methods and technological equipment are required to improve the community's traditional forest management ability. For example, when young indigenous people return to the community after spending some time living in cities, they may be unable to obtain accurate information about the community or its forest management measures quickly through life experience or oral history. This is because learning from life experience typically takes a long time, and the loss of information can occur during the passing on of oral history because of the differences in language use between the young and old members of the community. In addition, smoke signals, calling out, and wrapping ribbons around trees are all means through which messages are conveyed by community members. However, the messages conveyed through such means can be obscured by the distance or unclarity of the signals. With contemporary technological advancements, the community can improve the effectiveness of its forest management through contemporary scientific methods, equipment, and blockchain platforms.

1. Establishing a talent database blockchain platform for the Paiwan community development association: This step involves the convening of an implementation team, compilation of the skills of the community members, and appointment of members to appropriate positions on the basis of their skills to maximize their contributions to the community [33]. Therefore, skill-related information of the community members (e.g., education background, experience, expertise, and special skills) can be digitalized to enable the clear presentation of their credentials, which serves as the basis for their appointment to appropriate positions; the aforementioned processes are all completed online. The incorporation of these skill data into the blockchain facilitates bilateral communication and coordination with organizations that are looking to fill their job vacancies. For example, in the case of river trekking arrangements, digitalized data enable quick access to information about guides, river trekking sites, and safety instructions.
2. Creating a resource network through blockchains: This step involves the formation of a dense network comprising related organizations and the police and fire departments, and this is achieved through the incorporation of their data into a blockchain. The network allows for the real-time exchange of information, such that timely responses and support can be provided to ensure the safety of community members [34]. Accordingly, resource allocation and interconnections within a blockchain carry multiple meanings in various places. For project management in a blockchain website, arrangements must be made for all project activities and the resources required for each activity (to determine which activities should be advanced or delayed), with the aim of achieving project goals and minimizing the time required to complete resource-constrained activities [35].
3. Establishing an inquiry platform for the community: The incorporation of information about the Paiwan community into a website enables individuals to access real-time information about events and developments related to the community through their personal devices. An inquiry response platform should be established, and this platform should be supported by personnel who are dedicated to providing comprehensive responses to receive inquiries [36]. Hough and Spillan [36] suggested that effective crisis management can be realized by establishing a crisis team, analyzing loopholes, formulating strategies and plans, and evaluating the performance of plans. For tourism, a blockchain platform provides a high degree of convenience; however, human involvement is still required because a blockchain only provides general information, and personnel are required to respond to unanticipated situations. When travelers visit the community, they are expected to hike, hunt, and learn about mountainous plants in the forests, and human involvement is a necessary component for such a diverse itinerary because these travelers will make inquiries that require human responses during their trip [37].
4. Establishing a blockchain for crisis management: This step involves providing appropriate support and guidance at the project management level and establishing a risk management culture in relation to the overall organization, resources, and scheduling. During the project implementation process, high standards should be established for risk management, and connections should be made with related organizations while making continual improvements to the project and providing updates on its progress [38]. Data from Taiwan's Central Weather Bureau and strategic forest management organizations can be incorporated. For example, a blockchain can facilitate the prediction of typhoons, floods, and landslides [36] and enable project members to access all related information through their computers and phones.
5. Establishing a blockchain for transportation network information: This step involves providing multiple travel options by consolidating the available transportation options (i.e., Taiwan Railways, Taiwan High Speed Rail, and buses) for travelers in accordance with their travel plans [39]. To prevent road accidents on the Sisaumaqa Djalan Road (previous accidents were primarily due to human error) and ensure the safety of the shuttle vehicles that use it, comprehensive road safety instructions should be provided, investment in transportation infrastructure should be increased, and the physical and mental health of shuttle drivers should be monitored. All basic information on shuttle vehicles (e.g., age and maintenance status) and of their drivers (e.g., driving experience, predrive alcohol test results, and violation records) should be digitalized and uploaded to a transportation blockchain.
6. Establishing a blockchain with satellite images: Sensor technology advancements and the availability of high-solution satellite images have facilitated the monitoring of changes on the Earth's surface. However, the complexity of satellite images affects the accuracy of the classification of such changes. Thus, the identification of differences is crucial. To increase the change detection accuracy of an algorithm for the aforementioned types of image features, the effective detection of changes is required, and inaccurate classification must be minimized. Map information concerning changes in height is key to improving classification precision [40]. Accordingly, satellite images should be used to enhance the community's monitoring of changes in the forests; through the utilization of readily available aerial and fixed-point photography, the community can obtain information about the distribution of forests, the conditions of sightseeing spots, and the reproductive status of various species in real time. This information can then be incorporated into the community's blockchain platform to facilitate the implementation of subsequent response measures [41].
7. Establishing a blockchain for video surveillance equipment: In a technological environment where digital surveillance systems are ubiquitous and continuously producing large amounts of data, manual surveillance is required to identify human activities in the public realm. Meanwhile, smart surveillance systems that can identify normal and abnormal activities are urgently needed because they allow for the effective monitoring of images sent from cameras that are designed to capture abnormal activities; the implementation of these systems can alleviate the lack of surveillance personnel [42, 43]. Furthermore, the inclusion of these systems can enhance the community's control over the number of people entering the mountain and the entry of unauthorized personnel.

Green thinking has become a normal activity because all of the activities involved in green thinking are oriented toward sustainable development and are therefore conducive to environmental and social development [44]. Accordingly, with the support and appropriate application of scientific methods and technological equipment, green thinking can greatly benefit the community's tourism promotion and traditional forest management. Specifically, the traditional management methods of the community can be converted into stable data and information for the sustainable management of forests.

## 7. Conclusions and Recommendations

When the Paiwan community was an autonomous community, its forest management model was centered on not affecting the wildlife; all members of the community considered how their actions might affect forest sustainability before using any forest resources. Therefore, the community did not emphasize how they should protect forests; instead, the concept and practice of environmental protection were already integrated into the everyday lives of community members, and various taboos were established to deter members from violating the related rules.

After Japan and subsequently Taiwan imposed their authority over the Paiwan community, forest management shifted toward the use of resources, with the aim of maximizing deforestation. However, the clearing of forest lands exposed the soil and rocks on the mountains, such that the detrimental effects of extreme weather on the overall environment outweighed the economic benefits gained from deforestation. Therefore, the government implemented extreme measures (e.g., the establishment of protected areas and national parks) to provide strict protection and prohibit unauthorized entry with respect to these sites. Additionally, indigenous people were relocated from the mountains on which they had lived for hundreds or even thousands of years, which deprived them of their forest-dependent livelihoods, namely hunting, harvesting, and farming. The government took over the forest resources that originally belonged to these indigenous people and relocated them away from their territory; this government policy hurt the Paiwan community, which had long been an integral part of the forest ecosystem. The government assumed that the forest would soon be restored to its original state after the indigenous people are gone; it overlooked the large-scale landslides in the mountains and forests that were caused by the large-scale deforestation that it had ordered. In response to new consumer needs resulting from economic development, the local traditional farming model of the community has shifted toward the cultivation of highly profitable crops to maximize farming profits. The community's farming area was expanded excessively and flood control measures were inadequate, which reduced the resistance of their lands to extreme weather conditions and hence soil and rock erosion.

The protection of mountainous forests involves not just forests but all the flora and fauna that are found in them. The excessive reproduction of a species may create an ecological imbalance that is detrimental to the forest environment. From the perspective of human rights, the government should not have sacrificed the rights of the minority for the purpose of implementing national policies.

According to the results of the present study, effective forest protection is only possible if the Paiwan community returns to its traditional living model, which focuses on striking an ecological balance in the forest, emphasizes a sharing culture, and, most importantly, incorporates the use of contemporary technological equipment, information processing methods, and management methods and knowledge. For example, blockchain technology can help the community to manage forests, ensure forest sustainability, minimize deforestation, and enhance the tourism value of forests, thereby expanding the role of forests as a source of materials to encompass all the organisms that are found in them. Accordingly, forest protection should move beyond the conventional centralized strategy. Typically, the government can close off a forest area or subject it to stringent controls without considering in depth the specific needs of each mountain; this strategy has been proven to be ineffective. Therefore, protection policies must be customized for each forest through an in-depth understanding of its environment. Contemporary technologies should be used to informatize and digitalize all types of information and develop blockchains for various information-related purposes. This strategy considers all the organisms that live in forests, and it is a sign of respect for the indigenous communities who have been living in forests, their lifestyle of coexistence with the forests, and their self-management culture.

## Data Availability

Historical data were used to support this study.
